# Development of Cultural and Creative Industries and the Innovation of Packaging Design under the Background of Big Data

This article has been retracted.

**DOI:** 10.1155/2022/5622901

**Published:** 2022-08-18

**Authors:** Sisi Liu

**Affiliations:** School of Packaging Design and Art, Hunan University of Technology, Zhuzhou 412007, Hunan, China

## Abstract

In recent years, the strong growth of cultural and creative industries has led to its occupying an increasingly important position in the social economy. The inheritance and development of traditional art forms are one of the most important sources of materials for the cultural and creative industries. Product packaging is an important part of visual communication. Under the influence of the rapid development of cultural and creative industries, packaging design has a new development trend. In addition to satisfying basic functions such as protection and transportation, today's packaging design has also been endowed with some new connotations. The article analyzes the development status and outstanding problems of Chinese packaging design. Combined with the significance of cultural and creative industries to packaging design, innovative explorations were carried out on various elements in the process of packaging design. The study found that in the analysis of the contribution of cultural and creative industries to the economy, the cultural and creative industries of City A have been showing a growth trend since 2015. And among the design concepts of environmental protection, emotional attention, and integration of Chinese and Western design concepts selected in packaging design, more than 80% of consumers agree to integrate environmental protection concepts into packaging design. A total of 67% of the public are in favor of incorporating the concept of emotional care into the design. A total of 54% of the public agree with the design concept of combining Chinese and Western. Understanding the preferences of customers is beneficial to making packaging design a highlight of product sales.

## 1. Introduction

In the late 1990s, in such an information-based world, few countries in the world were able to clearly realize that a new way of development had emerged in the world, which cleverly connected culture and economy. The form of creative products based on cultural resources can actually change the future economic destiny of a country. The creative industry has also changed from a simple concept to a huge economic benefit, which is enough to affect the development of a country. Developed countries were the first to attract worldwide attention with their creative products, marketing, and services, and set off a wave of creative economy. All countries in the world are considering developing the cultural and creative industries in their own unique ways and fields. With the advent of the era of globalization, all countries in the world have begun to pay attention to the unique cultural factors of their own nation, realizing that the unique cultural factors of their own nation can develop their own cultural industries.

With the enhancement of brand strategic awareness, China has put forward new requirements for the development of cultural and creative industries. It requires innovation and development of well-known brands with independent intellectual property rights and competitiveness. On the other hand, many domestic companies ignore the importance of packaging and carry out extensive advertising campaigns, focusing only on adding value to branded products to strengthen their brand image. Today, economic globalization has led to increased competition among brands. Packaging design has become an important factor that cannot be ignored in improving the competitiveness of brands in international and domestic markets. All brands hope to create a good image and add value to their brand through excellent packaging design. The vigorous development of cultural and creative industries has a decisive impact on China's long-term strategic development. Because it cannot only enhance China's economic strength, cultural, and social value of packaging design, but also guide China's industrial development on a sustainable path.

This paper proposes big data to guide the practice of packaging design, takes big data as the research background, and raises the commodity packaging design under big data to a theoretical level. Based on the powerful information retrieval capabilities, fast information processing capabilities, and massive data analysis capabilities of big data, the application of big data in the commercial field makes online marketing precise and efficient. Therefore, it provides new ideas and design decision-making methods for commodity packaging design and promotes commodity packaging design to adapt to the development of the times.

## 2. Related Work

The cultural and creative industries have always been considered a field of high innovation. However, research into its renewal process is divisive and incomplete. Cristian reviewed the existing innovation literature in the manufacturing industry and proposed a scientific model of the whole innovation process. This model is based on the issues of pregnancy, development, prevalence, and the role of external factors. Essentially, it explains how innovation happens and what management practices are often used. This is the first study that explores the model for the whole process. Based on this recommendation, an idea for future research is proposed [1]. Those destinations that are more attractive to tourists are those countries, regions, and places that offer the highest value for the money invested or those that offer uniqueness and exclusivity that cannot be replaced by other destinations. The aim of Jovii–Vukovi et al. was to point out the possibilities, significance, and synergies of the cultural and creative industries in the branding of tourist destinations. Research methods include cabinet research, a review of selected scientific and professional literature, and a presentation of local best practices. These places promote the development of innovative tourism through the recognition and affirmation of the creative industry, thereby ensuring their economic prosperity and image enhancement [2]. Calignano and Josendal's study contributed to limited literature. The study aims to examine the type and frequency of links between production facilities and higher education institutions (HEIs). The purpose of the study was to investigate the extent to which many types of links contribute to improving the innovation capacity of creative companies. Energy analysis shows that higher education institutions are not always closely linked, as other factors play a specific role in innovation potential. As explained and discussed, this finding depends to a large extent on some of the particular characteristics of the university, the technical perspective (basic knowledge) used by the construction companies, and the cultural differences between the two places [3]. Mao described the concept and characteristics of culture and the manufacturing industry in the digital economy and analyzed how culture and the manufacturing industry development in the digital economy. The cultural and creative industry during the digital economic system is based on a combination of Chinese culture and digital technology and creative technology, based on the creative knowledge of individuals or companies. In today's digital economy, the culture and manufacturing industries are innovative, cost-effective, and networked. The report also briefly analyzes the current challenges facing the cultural and creative industries. Mao proposed the protection of intellectual property rights for cultural and creative companies and the development of policies and practices for the management of cultural and creative companies to secure their place in the global market for culture and creativity. But it is not very practical [4].

With the enhancement of brand strategic awareness, China has put forward new requirements for the development of cultural and creative industries. It requires innovative development of well-known brands with independent intellectual property rights and competitive strength. How to innovate brand packaging design in this new era of cultural and creative industry development is a hot research topic at present. Carlin researched the “27th Tokyo Packaging Fair,” which took place from October 2 to 5, 2018. It offers a wealth of ideas, materials, products, and technologies for packaging designers, engineers, application engineers, and visual effects enthusiasts. The event, held at the Tokyo Ariake Convention Center in Ariake, Tokyo Bay, attracted more than 700 exhibitors, mostly from Asian countries, with Japan providing the largest number of participants [5]. Joachimiak–Lechman et al. presented a two-dimensional comparison of laminate alternative manufacturing processes in packaging for the food industry. The main objective was to evaluate the possible environmental impact during the production of two-layer laminates comprising the patented polypropylene film Metallyte 28UBW-ES, as well as the pap/LDPE/Al/LDPE multilayer laminates used to date. The environmental assessment is complemented by a cost calculation, which specifically takes into account the investment required to produce a two-layer laminate. In the study, life cycle assessment and life cycle costing methods were applied. Performance indicators are determined based on the environmental impact indicators obtained and the reduced costs. The results of the comparative analysis are displayed on a two-dimensional ecosystem activity map. According to the study, it was found to be prudent to replace traditional packaging materials with sheets containing the Metallyte 28UBW-ES system. A higher traffic rate may indicate this. The discrepancy between the production processes analyzed is small. However, in terms of environmental impact, support for double-layered sheets is a normal deficit [6]. The abovementioned studies have carried out a detailed analysis of the application of virtual interaction technology. It is undeniable that these studies have greatly promoted the development of the corresponding fields. Much experience can be learned from methods and data analysis. However, there are relatively few studies on the development of cultural and creative industries and packaging design by big data technology. It is necessary to fully apply these techniques to research in this field.

## 3. Integration and Innovation of Cultural and Creative Industry Development and Packaging Design under the Background of Big Data

There are broad and narrow definitions of construction companies. The wider creative economy refers to the cultural and creative industries. A narrowly created economy refers to a number of different companies and sectors that use creative knowledge for research, development, manufacturing, and marketing [7]. It is a new concept, a way of thinking and planning created within a global community of users. It encourages innovation and individual creativity and focuses on supporting and promoting culture and the arts in business. The key points for creative industries are as follows.

### 3.1. Compatibility

The core of the creative economy is creativity, and the basis of creativity is the fusion of different human disciplines. Disciplinary movements alone cannot generate sustainable creativity [8]. The basic idea of the creative economy is to promote “cross-border” reorganization and cooperation of different sectors and fields. It promotes cultural and economic development by transcending borders and seeking new growth points.

### 3.2. Collaborative

Originality is crucial in the creative industries, but it cannot be done behind closed doors by individuals. The creative industry is a chain industry that relies on the cooperation of creative teams, including creative design, creative planning, creative research and development, creative production, creative management, creative marketing, and many other links [9].

### 3.3. Copyright Awareness

Copyright protection is the oxygen on which the creative industries depend. Because the creative industries are industries built on creativity and individual skills and talents. It is possible to create wealth and increase efficiency by creating and acquiring intellectual property. The development of construction companies is inseparable from the protection of intellectual property rights and intellectual property rights are the foundation of the cultural and creative industries. The success or failure of copyright development in a country or region depends directly on the completeness of copyright protection [10].

Cultural industries can be divided into core sectors of creative arts, other core sectors of cultural industries, extended cultural industries, and related industries, as shown in Figure 1. The core sectors of the creative arts include culture and arts, printing and publishing, radio, television and film, and the art trade. Other major cultural industries include advertising and exhibition services, design services (fashion design, interior design, and graphic design), architecture and software, and network and computer services [11]. The broader cultural industry includes tourism, leisure, and entertainment services. Core cultural and creative industries refer to industries that focus on cultural and creative content, products, and services related to intellectual consumption. Regional cultural industries are industries that provide cultural and creative services to other industries. The production of cultural and creative industries requires a certain degree of creativity. The related industries are mainly auxiliary services for the production and sale of cultural products and cultural equipment [12].

While the cultural and creative industries bring wealth and employment growth to society, it is more important to promote cultural diversity, social development, and human development [13]. Characteristics of cultural and creative industries:

#### 3.3.1. Profound Cultural Concept

The cultural and creative industries usually have two content sources: one is the content developed by creativity and innovation based on traditional culture, and the other is the new cultural content developed by contemporary creativity and innovative ideas [14]. Whether traditional or modern, transformational or creative, cultural concepts are the main content of the cultural and creative industry and the most important factor in its development. Likewise, the economic development of modern society has undergone major changes. Because it has become both an economic form and a cultural phenomenon. Culture can greatly contribute to economic development. It can be seen that the development of sustainable development is inseparable from traditional culture, and the connotation of traditional culture is also an important material reserve for sustainable development [15]. The main content of the output of cultural and creative industries originates from traditional culture and is different from traditional culture. The essence is the creative development and utilization of traditional cultural resources and cultural concepts, and the inheritance and development of traditional culture in modern society. Only when traditional cultural concepts are integrated into the cultural and creative industries can they have taste, value, and competitiveness.

#### 3.3.2. Wide Application of Modern Scientific and Technological Achievements

In addition to the innovative development of traditional culture, the emerging scientific and technological achievements in modern society are also widely used by the cultural and creative industries. This is not only the embodiment of its characteristics of the times but also the main means of its innovation [16]. Taking information and network technology as an example, it has now become one of the main carriers of cultural and creative industries. This also enables the deep integration of scientific and technological achievements with the development of contemporary culture. At present, many people in the industry are emphasizing that cultural accumulation and technological development are the main sources of creativity. Therefore, they pay more attention to the use of the latest technological achievements and means of expression in their creativity. Therefore, the extensive application of modern scientific and technological achievements is another main feature of the cultural and creative industries. It is one of the means for the overall development of the industry, such as the widespread application of the virtual reality technology commonly used in the cultural industry in the Shanghai World Expo, which reflects this feature [17]. It can be seen that the development of the cultural and creative industries has largely benefited from the extensive application of modern scientific and technological achievements, which has also greatly enhanced the influence of the cultural and creative industries.

#### 3.3.3. Characteristic Business Operation Model

Different from the traditional manufacturing products, the products, and services of the cultural and creative industries have a distinctive business operation mode. This model got rid of the past production-centered form and turned to emphasize the rendering of cultural ideas, the realization of creative works, and increased publicity and promotion [18]. This is particularly evident in the successful commercialization of Disney in the United States. The two cartoon characters “Mickey Mouse and Donald Duck” created by Disney Company were first made into cartoons and won the love of people. It took this as an opportunity to endow them with unique cultural attributes so that the derivative products produced by these cartoon images extended to clothing, toys, entertainment, and other fields. This enables the original independent cartoon image individual to develop a complete animation industry chain, laying the foundation for Disney to become a multinational group [19]. It can be seen from this real case that another characteristic of the cultural and creative industry is the adoption of a brand-new business operation model of “creativity + technology + capital.” That is to say, based on an excellent idea, a unique culture has been developed. Then, through advanced scientific and technological means, the virtual cultural concept is transformed into real products, and then the operation mode of the industrial chain is improved to open up a wider market [20].

The development of cultural industries should be assessed in three dimensions: cultural assets (capital), infrastructure and policy frameworks, and cultural production (products and services) [21]. The theoretical basis of the framework construction, the selection of measurement variables, and the construction of the Chinese provincial and municipal cultural industry development index system model are shown in Figure 2.

The cultural and creative industry indicator system consists of cultural and creative industry input indicators, cultural and creative achievement output indicators, and policy support. Cultural and creative capital investment indicators are composed of three categories of indicators, namely cultural capital, creative capital, and human capital. It can reflect the development potential of cultural and creative industries in the region, as shown in Figure 3. The output indicators of cultural and creative achievements are three types of indicators that can reflect the development level and status quo of cultural and creative industries in the region, including cultural and creative products and services, international trade, and output scale.

With the passage of time and the continuous advancement of technology, people's living standards have been greatly improved. With the continuous segmentation of the market and the improvement of consumer awareness, the traditional single sales packaging can no longer meet the needs of consumers, and the creative and attractive packaging has gradually won personalization. Today's packaging design not only implements basic protection and transportation functions but also employs some new concepts. Personal clothing cannot only enhance the brand and promote sales but also meet the emotional needs of consumers and inhibit consumers' sensory experience and inner psychological pleasure [22, 23].

Internet-based online shopping platforms and rapidly developing big data technology are collections of information about big data. The company collects vast amounts of data about businesses, products, competitors, and consumers via the Internet, analyses and processes the data, relates commercial value, and facilitates the marketing of personal pressure [24, 25]. The online shopping market is very competitive. As one of the important competitive advantages of raw materials, big data also play an important role in the packaging design of raw materials. Research on raw material packaging design through a large database can inspire methods and ideas for raw material packaging design [26, 27].

The design process of the big data mining system includes data collection, data preprocessing, mining model construction, and mining model visualization, as shown in Figure 4.

1. Data collection: it mainly integrates databases according to the objects to be extracted, determines the size of the extracted database, eliminates data noise, and eliminates blank records and records with empty fields [28, 29].
2. Data preprocessing: it processes the data collected by monitoring to ensure the authenticity of the data. It is merged with the original database and deleted, and the data format is converted to meet the processing requirements of the association rule extraction system.
3. Building a mining model: in a mining system, one or more data mining methods can be used for data analysis and generalization. It mines the various rules, patterns, and trends that users need.
4. Mining model viewing: the system uses the optimized association rule mining algorithm to mine the information required by users. The mined rules will be saved in the knowledge base, which can be used for further analysis and use of the data in the future.

The big data mining system mainly includes the overall design of the system and the design of each function of the system, each function of the system: data source selection module, data preprocessing module, transformation data module, output and visualization of association rules, etc., as shown in Figure 5.

Cluster analysis and association rules are two types of mining problems in the big concept of data mining. Cluster analysis is the unsupervised discovery of clustering effects among data. Association rules are the statistical discovery of potential connections between data. Clustering can be understood as the process of dividing a dataset into groups or clusters of similar objects. Thereby, the similarity between objects in one group is maximized, and the similarity between objects in different groups is minimized. There are only two cores of cluster analysis methods, one is the similarity measurement of samples, and the other is the problem of clustering criteria. Clustering methods include statistical analysis methods, machine learning methods, neural network methods, etc. The results of cluster analysis can be used to understand customer preferences and bring economic benefits. The purpose of cluster analysis is to mine useful patterns or knowledge in a large amount of potentially useful data. Cluster analysis is based on similarity. There are more similarities between patterns in one cluster than patterns not in the same cluster. How the data are stored is also a critical issue. There are two common data structures for clustering algorithms.

(1)   Data matrix: a data matrix is actually a relational table. A row in a matrix represents a data object. A column in the matrix represents an attribute of the object. Supposing there are *q* objects, *C*=(*c*_1_, *c*_2_, ..., *c*_*n*_), in the dataset, and each object has *p* attributes. Then this relational table can be represented as a *q *×* p* matrix:
  (1) $$\begin{array}{c} \left(\begin{array}{ccc} c_{11} & \ldots & c_{1p}\\ \ldots & \ldots & \ldots \\ c_{q1} & \ldots & c_{qp} \end{array}\right). \end{array}$$
Among them, *c*_*ij*_ represents the jth attribute value of the data object *c*_*i*_, 0 < *i* < *q*, 0 < *j* < *p*.
(2) Difference matrix:

The difference matrix is an *n *×* n* dimensional matrix that stores the dissimilarity between objects. Among them, the element *a*(*i*, *j*) represents the dissimilarity between objects *i* and *j*. It is expressed as follows:

(2) $$\begin{array}{c} \left(\begin{array}{ccccc} 0 & \; & \; & \; & \;\\ a\left(2,1\right) & 0 & \; & \; & \;\\ a\left(3,1\right) & a\left(3,2\right) & 0 & \; & \;\\ \ldots & \ldots & \ldots & \ldots & \;\\ a\left(n,1\right) & a\left(n,2\right) & \ldots & \ldots & 0 \end{array}\right). \end{array}$$

In general, *a*(*i*, *j*) is a non-negative number. The smaller the value, the more similar entity *i* and entity *j* are. In cluster analysis, the data structure is mostly used in the form of a different matrix. If the data is given in the form of a data matrix, it is often necessary to convert the form of the data matrix to a different matrix.

In cluster analysis, in order to eliminate the influence of size differences on clustering results, it is usually necessary to normalize data attributes before clustering. It converts various dimensions into normalized dimensionless measures. Supposing there are *n* data objects in the dataset:

(3) $$\begin{array}{c} X=\left(b_{1},b_{2},\ldots ,b_{n}\right). \end{array}$$

Each data object has *m* attributes, that is, the data matrix corresponding to *c*_*i*_=(*c*_*i*1_, *c*_*i*2_,…, *c*_*im*_):

(4) $$\begin{array}{c} A=\left(\begin{array}{ccc} c_{11} & \ldots & c_{1p}\\ \ldots & \ldots & \ldots \\ c_{q1} & \ldots & c_{qp} \end{array}\right). \end{array}$$

Among them, *c*_*ij*_ represents the jth attribute value of data object *c*_*i*_, 0 < *i* < *q*, 0 < *j* < *p*.

Common data specification standard methods are as follows:

(1) Standard deviation normalization:
  (5) $$\begin{array}{c} c_{ij}=\frac{c_{ij}-{\bar{c}}_{i}}{\mu_{j}}. \end{array}$$
Among them,
  (6) $$\begin{array}{c} {\bar{c}}_{i}=\frac{1}{n}\sum_{j=1}^{p}c_{ij}, \end{array}$$
where ${\bar{c}}_{i}$ represents the mean of data object *c*_*i*_,
  (7) $$\begin{array}{c} \mu_{j}=\sqrt{\frac{1}{n-1}\sum_{i=1}^{q}{\left(c_{ij}-{\bar{c}}_{j}\right)}^{2}}, \end{array}$$
where *μ*_*j*_ represents the standard deviation of the data sample on attribute *j*.
(2) Maximum value normalization:
  (8) $$\begin{array}{c} c_{ij}^{\prime }=\frac{c_{ij}}{c_{j_{\max}}},\\ c_{j_{\max}}=\max\left\{c_{1j},c_{2j},\ldots ,c_{nj}\right\}, \end{array}$$
where *c*_*j*_max__ represents the maximum value of the data object on the attribute *j*.
(3) Mean normalization:

(9) $$\begin{array}{c} c_{ij}^{\prime }=\frac{c_{ij}}{{\bar{c}}_{j}}. \end{array}$$

Among them,

(10) $$\begin{array}{c} {\bar{c}}_{j}=\frac{1}{n}\sum_{i=1}^{n}c_{ij}. \end{array}$$

It represents the mean of the data object on property *j*.

The dissimilarity coefficient between two objects is a numerical measure of how different two objects are. Common similarity coefficients are as follows:

(1)   Cosine of the included angle: The cosine of the angle between two vectors can be used to represent the similarity coefficient. Its similarity coefficient is as follows:
  (11) $$\begin{array}{c} s_{ij}=\cos\left(\alpha_{ij}\right)=\frac{\sum_{k=1}^{p}x_{ik}x_{jk}}{\sqrt{\sum_{k=1}^{p}x_{ik}^{2}\sum_{i=1}^{p}x_{jk}^{2}}}. \end{array}$$
(2) Correlation coefficient:

The correlation coefficient between data objects *x*_*i*_ and *x*_*j*_ has the following expression relationship:

(12) $$\begin{array}{c} r_{ij}=\frac{\sum_{k=1}^{p}\left(x_{ik}-{\bar{x}}_{i}\right)\left(x_{jk}-{\bar{x}}_{j}\right)}{\sqrt{\sum_{k=1}^{p}{\left(x_{ik}-{\bar{x}}_{i}\right)}^{2}\sum_{k=1}^{p}{\left(x_{jk}-{\bar{x}}_{j}\right)}^{2}}}. \end{array}$$

Among them, ${\bar{x}}_{i}$ and ${\bar{x}}_{j}$ are the mean values.

(13) $$\begin{array}{c} {\bar{x}}_{i}=\frac{1}{p}\sum_{k=1}^{p}x_{ik}. \end{array}$$

Apriori algorithm is the first and most classic association rule mining algorithm. It uses an iterative search method based on a layer-by-layer search to find relationships between item sets in the database to form rules. The process includes concatenation (operations on class matrices) and pruning (removal of unwanted intermediate results). The Apriori algorithm adopts an iterative method of layer-by-layer search. The algorithm is simple and clear, without complicated theoretical derivation, and easy to implement. The association rule extraction problem can be divided into two subproblems.

1. In the transaction database, it searches for all frequent item sets greater than or equal to user-defined minimum support.
2. It uses frequent item sets to generate all association rules, chooses according to the minimum confidence specified by the user, and finally obtains strong association rules. That is, for any set of frequent elements L and any nonempty subset *S*⊆*L* of L, if the ratio

(14) $$\begin{array}{c} \frac{\text{Support}\left(L\right)}{\text{Support}\left(S\right)}\geq \text{minconf,} \end{array}$$

then generate valid association rules as

(15) $$\begin{array}{c} R:S\Rightarrow \left(L-S\right). \end{array}$$

And the confidence and support of the rule are

(16) $$\begin{array}{c} \text{Confidence}\left(R\right)=\frac{\text{Support}\left(L\right)}{\text{Support}\left(S\right)},\\ \text{Support}\left(R\right)=\text{Support}\left(L\right). \end{array}$$

Most cultural and creative enterprises are committed to presenting traditional Chinese culture in the product packaging design but are also exposed many problems. For example, the design concept is too traditional to keep up with the pace of international design concept updating, and the market positioning is not clear. In order to highlight local characteristics, some packaging designs fabricated some ethnic representative patterns out of thin air or appeared to be wearing a crown and wearing a hat without research. Some do not consider the visual characteristics of domestic consumers at all and copy the design styles of Japan and some western regions, and the results are mediocre. These are all caused by the design concept entering misunderstanding. When you buy tea, you will find that there is a dazzling array of tea products, and most of them have the same packaging. Whether it is the shape, color, material, or packaging form of the packaging, they are very similar. Consumers cannot tell the difference at all and even doubt whether there are fakes, and there is no sense of human touch and design. There is also the phenomenon of overpackaging such as “gold and jade in the outside, ruin in the middle.” It blindly pursues the external gorgeous packaging effect. It looks very refined and looks high-end. The products inside are indeed uneven, and some are even ranked second. These packaging designs that deviate from the essence of the packaging are not recommended.

The influence of cultural and creative industries on packaging design is mainly reflected in two aspects: the influence on packaging design concepts and the influence on packaging design media. On the one hand, from the perspective of the development of cultural and creative industries, packaging design should shift from purely functional load to cultural creativity. Packaging design should pay more attention to the expression of cultural connotation so that users can perceive the corresponding relationship between packaging and products in the cultural connotation. On the other hand, it starts from creativity and cultural creativity and implies new requirements, that is, it refuses to systematically apply traditional cultural elements to packaging design support, but adopts new methods and design techniques. Instead, culture must be reinterpreted with new design methods, techniques, and structures. With the development of cultural and creative industries, the innovation of packaging design can be reflected in the following aspects: it intelligently arranges elements such as text, logos, graphics, and colors to enhance the visual effect of packaging. It carries out cultural and creative packaging design on packaging materials, such as paper, glass, metal, and wood. The different textures and proposals of the material itself add a special aesthetic. Different textures and suggestions of the same material bring different psychological, as well as visual and tactile sensations to product packaging. Common packaging structures mainly include wall, sky and Earth cover, swing cover, and window opening. Depending on the existing structure, combined with the principles of protection and convenience of packaging design, creative window design or special-shaped design is carried out on the structure according to the characteristics of graphics or text. For example, the packaging structure is made closer to it with the elements of local building forms or typical cartoons, or even a certain theme. Graphics and text can be placed creatively according to the structure. At the same time, considering the interconnection of products, the design of packaging series of different structural forms can be made consistent. Finally, it is also possible to select structures related to product characteristics. This not only reflects the characteristics of the product but also creates a sense of familiarity.

1. Promote national culture and pay attention to the inheritance of local culture.
2. National culture is the sum of material and spiritual wealth that fully reflects the characteristics of the nationality, produced and created by the people of all nationalities in the long-term common production and life activities including philosophy, literature, folklore, and art. To carry forward the national culture is not to simply copy the classical culture, but to have a deep understanding of the national culture and grasp the essence of the national culture on the surface. Only by grasping the form can it grasp the essence of national culture.
3. Focus on the leadership of consumer culture.

Consumption culture is only the sum of the consumption concept, consumption method, consumption behavior, and consumption environment that people show in consumption activities. Faced with consumer groups of different nationalities, classes and cultures, because they live in different social and cultural conditions, they have different aesthetics for product packaging.

## 4. Cultural and Creative Industry Development Data Retrieval Experiment

Distributed File System (HDFS) is one of the core technologies of Hadoop, which can store and manage massive data in a distributed manner. When data are loaded into HDFS, the master node manages file access for each node, as shown in Figure 6.

In order to study the time performance analysis of the data retrieval system, 14 Ultra-TR227 servers of Tsinghua Tongfang were used in the experiment. A cluster of nine nodes participated in the experiment, with one node serving as the NameNode (master) and the other eight nodes serving as DataNodes (slaves), with the same interface as the nodes. In the experimental machine, the Linux operating system is installed under Windows using a virtual machine. This enables the Hadoop operating environment. The data used is stored in files with a support degree of 0.7, and 8 data nodes in the cluster are used for testing. The results are shown in Table 1.

It can be seen from Table 1 that when the amount of data is not large, the MR-Apriori algorithm based on the map-reduce framework under the Hadoop platform is not significantly different from the traditional Apriori algorithm. But as the amount of data increases, it takes longer to try. As can be seen from the analysis, the reason for this phenomenon is that when the amount of data is small, the proportion of time spent in network communication is higher. When the amount of data increases, the proportion of time that the system processes the data increases, and the time for network communication can be ignored. The following experiments on synchronous data processing in a cluster environment show that in a big data environment, MR-Apriori is more suitable for processing large amounts of data than traditional Apriori. And as the amount of data increases, the efficiency of MR-Apriori compared with independent processing becomes more and more obvious.

In the experiment, data volume 1 (100, 300, 500) and data volume 2 (300, 500, 800) are called, respectively, and 2, 4, and 8 nodes are called for map processing. The results are recorded in Table 2.

## 5. Development Status of Cultural and Creative Industries and Innovative Direction of Packaging Design

The economic value created by the cultural and creative industries has become an important pillar of the national economy. The development of cultural and creative industries objectively shows that increment (new industry) exceeds stock (traditional industry) and technology promotes the development of industrial increment. The cultural and creative industry has the development characteristics of rapid growth in total volume, continuous optimization of the structure, increasingly rational layout, distinctive regional characteristics, and outstanding industrial advantages. The industrial development model has been fundamentally shaped, and the industrial service system has been gradually improved. Their status as a pillar industry of the regional economy has become more and more stable, and stimulated the development of many surrounding industries, thus becoming a new pole of economic development. In order to study the empirical evidence of the contribution of the cultural and creative industries to the economy, it chooses to analyze the development of the cultural and creative industries in City A in recent years.

Figure 7 shows the results of the dynamic analysis of the culture and manufacturing industries in City A. In this way, the direct impact of culture and manufacturing industries on the contribution of the system is a study.  Figure 8 is an analysis of the economy's contribution to economic culture and industry.

As can be seen from Figure 7, the cultural and creative industry has been showing a growth trend since 2015. Software, network and computer services, news and publishing, radio, television, and film industries are growing rapidly and have a large proportion. In particular, the added value of software, network, and computer services will account for 50% of the added value of the cultural and creative industries in 2020. They are the city's strengths and focus industries.

As can be seen from Figure 8, the relative growth rates of the cultural and creative industries in City A and the overall economy both exceeded 1. It shows that the growth rate of cultural and creative industries exceeds that of the overall economic situation, which supports the growth model. From 2015 to 2020, the relative growth rate of the cultural and creative industries to the overall economy will reach more than 1.2. In 2018, the relative growth rate of cultural and creative industries reached 2.4. The growth rate of cultural and creative industries to overall employment is as high as 1.5 or more. The effect of cultural and creative industries on employment growth is particularly significant. In order to study the influence of packaging design factors on the purchase intention of citizens, the article randomly selected 100 ordinary citizens as the survey objects, including 50 males and 50 females. The basic information of the experimental subjects is shown in Table 3.  Figure 9 shows the results of a survey on citizens' preference for product packaging design.

It can be seen from Figure 9 that the age factor has a big difference for citizens in the choice of product packaging design. The respondents under the age of 30 were mainly selected based on two factors: the individualization of product packaging design and product quality. Among them, 26 people choose personalized packaging design factors.

The design concept innovation of packaging mainly has three aspects: the design concept of environmental protection, the design concept of emotional concern, and the design concept of integration of Chinese and Western. In order to study the tendency of consumers toward the three concepts, 100 respondents were specially asked for different opinions on the symbol. The results are shown in Figure 10.

As shown in Figure 10, more than 80% of consumers are in favor of incorporating environmental protection concepts into packaging design. Excessive packaging brings unnecessary waste of resources to society, increases the cost of enterprises, and also brings unnecessary expenses to consumers. Consumers from the 1980s and 1990s are now the largest consumer group. They usually have stable incomes and higher educations and are able to keep up with the times. Today, the desire for simplicity and style is a major consumer trend for this group. The research results demonstrate the feasibility and superiority of the eco-design concept. A total of 67% of the public support incorporating the concept of emotional care into the design. With the development of science and technology and productivity, people's material life has been greatly improved, and more and more people are beginning to pursue spiritual satisfaction. The style is modern and novel, with a strong sense of modernity and movement, which meets the emotional expectations of most young consumers, making this product series quickly accepted by consumers. Only 54% of the public support the design concept of combining Chinese and Western, because some packaging lacks modernity, the use of technology is too cumbersome and relies on modern Western design concepts and technologies. The essence of traditional Chinese culture must be incorporated into the concept of modern Western design. This is not simple addition, but a fusion based on a deep understanding of Chinese culture.

## 6. Conclusion

Based on modern packaging design theory, this paper conducts research and analysis to guide the current situation of packaging design at home and abroad. To sum up, modern packaging design has been impacted by the cultural and creative industries and has a new development trend. The cultural and creative industry can only form an industry based on “culture,” and the development of the industry has become the driving force for the continuous progress of packaging design. With the development of economic globalization, brand packaging design has not only become the leader of the creative industry but also an important part of it, and has a position that cannot be ignored. Packaging is no longer simply used to preserve and protect items. Modern packaging has risen to a new height, not only can convey the basic information and attributes of commodities but also contains the profound cultural heritage, which is a double aesthetic enjoyment of vision and spirit. The injection of cultural elements is also a clear spring to highlight the personality of the packaging. Only packaging with profound cultural connotations is fresh and alive. In the context of cultural and creative development, brand packaging design has a more long-term and broad development prospect. It cannot indulge in the past packaging design management. Now is the age of information technology, and it should be learned from design masters. It not only learns to learn from its excellent design concepts and design methods but also adds its own innovation, and strives to surpass the masters instead of imitating them.

## Figures and Tables

**Figure 1:** Criteria for the division of cultural and creative industries.

**Figure 2:** Construction of China's provincial and municipal cultural industry development index system model.

**Figure 3:** Framework for the establishment of evaluation indicators for cultural and creative industries.

**Figure 4:** Data mining process.

**Figure 5:** System functional structure diagram.

**Figure 6:** The architecture of HDFS.

**Figure 7:** The added value of cultural and creative industries in 2015–2020.

**Figure 8:** Analysis of the contribution of cultural and creative industries to the economy.

**Figure 9:** Survey results of citizens' preference for product packaging design.

**Figure 10:** Survey results of consumers' preference for three concepts.

**Table 1:** Test results.

Data volume (million)	1	5	10	50
Single machine (sec)	110	121	145	271
2 nodes (seconds)	185	199	282	835
4 nodes (seconds)	156	164	261	492
6 nodes (seconds)	152	158	235	432
8 nodes (seconds)	145	155	228	400

**Table 2:** Processing efficiency.

Mode	Data volume 1	Data volume 2
Stand-alone	1	1
2 node machines	0.26611	0.79562
4 node machines	0.18659	0.38659
8 node machines	0.11425	0.22554

**Table 3:** Basic information of the respondents.

		Males	Females
Age	≤15	10	8
	16–30	22	20
	31–45	12	17
	≥45	6	5

## Data Availability

Data sharing is not applicable to this article as no new data were created or analyzed in this study.
